# Expression and Clinical Significance of HER2 Gene and DNMT1 in Non-Small-Cell Lung Cancer

This article has been retracted.

**DOI:** 10.1155/2022/8426384

**Published:** 2022-08-13

**Authors:** Weiying Diao, Chenglong Ding, Boyang Yuan, Zan Li, Na Sun, Jiabin Huang

**Affiliations:** ^1^Department of Pathology, The First Affiliated Hospital of Jiamusi University, China; ^2^Department of Acupuncture and Mimoxibustion, The First Affiliated Hospital of Jiamusi University, China; ^3^Department of Analytical Chemistry Teaching and Research, Jiamusi University, China; ^4^Graduate Department, Jiamusi University, China; ^5^Department of Geratology, The First Affiliated Hospital of Jiamusi University, China

## Abstract

**Objective:**

To explore the expression and clinical significance of HER2 and DNMT1 in non-small-cell lung cancer.

**Methods:**

The patients with non-small-cell lung cancer treated in the First Affiliated Hospital of Jiamusi University between 2018 and 2020 were enrolled in this study. The serum DNMT1 concentration and the expression of HER2 protein in lung cancer and adjacent tissues of the two groups were analyzed.

**Results:**

The DNMT1 protein concentration was significantly correlated with gender, age, and smoking history of patients. HER2-positive expression was significantly related to tumor type, tumor size, tumor differentiation degree, and lymph node metastasis. However, HER2 levels were not related to the gender and smoking history of patients.

**Conclusion:**

High expression of DNMT1 protein in serum may increase the risk of non-small-cell lung cancer and may play an important role in the early development of lung cancer. HER2-positive expression may promote the development of advanced and metastatic non-small-cell lung cancer.

## 1. Introduction

The incidence and mortality of lung cancer ranks first among tumors, of which about 85% are non-small-cell lung cancer (NSCLC) [1, 2]. Due to the high degree of malignancy, the 5-year survival rate was only 18.4%. Epidermal growth factor receptor 2 (HER2) and human epidermal growth factor receptor 3 (HER3) belong to the receptor tyrosine kinase (RTK) superfamily, both of which can produce heterodimers to participate in tissue signal transduction, endangering cell differentiation, erosion, differentiation, and migration [3, 4]. DNA methyltransferase 1 (DNMT1) is the most abundant methyltransferase in cells, and its role is to maintain DNA methylation [5, 6]. The abnormal expression of DNMT1 and HER2 genes may cause the loss of tumor suppressor gene function and the increase of protooncogene activity, which play a key role in the development trend of various malignant tumors [7]. The purposes of this study were to investigate the expression and clinical significance of HER2 gene and DNMT1 in non-small-cell lung cancer and to provide a theoretical basis for the mechanism research and antitumor research of non-small-cell lung cancer.

## 2. Materials and Methods

### 2.1. General Information

From 2018 to 2020, 60 patients with non-small-cell lung cancer in the First Affiliated Hospital of Jiamusi University were selected as the observation group. The control group consisted of 60 normal people who underwent physical examination during the same period. The patient informed consent to this scientific research and this study was approved by the hospital ethics committee.

### 2.2. Detection of DNMT1 Protein Concentration in Serum

The DNMT1 protein concentration in serum was determined by DNMT1 ELISA Kit (ab113469, Abcam, USA) following the manufacturer's instructions.

### 2.3. HER2 Protein Expression in Lung Cancer and Adjacent Tissues

The collected specimens were fixed with 10% formalin for 12 hours, then embedded in 4 *μ*m thick paraffin sections, and smoked at 68°C for 1-1.5 hours. The paraffin section specimens were collected. After deparaffinization and solidification, the endogenous peroxidase solution was blocked with 3% hydrogen peroxide, and the rabbit anti-human HER2 antibody (MA5-13675, Invitrogen, USA) was incubated for 0.5 h at 37°C and overnight at 4°C. The Goat anti-Human IgG Secondary Antibody (A18817, Invitrogen, USA) was incubated at 37°C for 1 h, developed with DAB, counterstained with hematoxylin, and mounted. Positive expression was brown and tan cytoplasmic staining; optical Image-Pro-Plus 6.0 image analysis software was used to analyze the expression of HER2 protein. The standard was used to score the color intensity and the number of color-developing cells [8]. The number of positive cells in 5 random fields of view was scored under a high-power microscope as follows.

The staining intensity was scored as 0, with no positive staining. 1 point, weak staining. 2 points, moderate staining. 3 points, strong positive staining. The percentage of positive cells was scored as 0, no positive cells. 1 point, the positive rate is less than 10%. 2 points, the positive rate is greater than 10% and less than 50%. 3 points, the positive rate is greater than 50%.

### 2.4. Statistical Methods

SPSS25.0 was used for statistical analysis. Data were presented as mean ± standard deviation (SD) and analyzed Student's *t*-test. *P* value less than 0.05 was considered statistically significant.

## 3. Results

### 3.1. General Information

The male/female ratio of patients in the observation group was 41/19, and the age structure was 60.43 ± 1.63 years old, 44 smokers and 16 nonsmokers. Histologically, 24 cases were squamous cell carcinoma, 19 cases were adenocarcinoma, and 17 cases were large cell lung cancer. The clinical TNM stage was 23 cases of stage I, 11 cases of stage II, 15 cases of stage III, and 11 cases of stage IV. In the control group, the male/female ratio was 39/21, and the age was 60.25 ± 1.49 years, 46 smokers and 14 nonsmokers. There were no significant differences in gender, age, and smoking history between two groups (*P* > 0.05, Table 1).

### 3.2. Comparison of DNMT1 Protein Concentration in Serum between Two Groups

As shown in Table 2, the patients in each group were divided based on gender, age, and smoking history. Compared to patients in control group, the DNMT1 concentration in observation group was significant higher in each category. The only exception was patients with smoking history; no significant differences were observed between two groups.

### 3.3. The Relationship between the Different Clinicopathological Characteristics and the Serum DNMT1 Protein Concentration

The relationship between different clinicopathological characteristics and serum DNMT1 protein concentration was analyzed. The serum DNMT1 protein concentration of NSCLC patients was significantly correlated with histological type (*P* < 0.05), and the serum DNMT1 protein concentration of patients with clinical stage I+II was significantly higher than that in stage III+IV (*P* < 0.05) (Table 3).

### 3.4. Expression of HER2 in NSCLC and Its Relationship with Clinicopathological Parameters

HER2 positivity is mainly expressed in the cell membrane and cytoplasm, and a small number of cells are expressed diffusely in the cell membrane, showing uniform brown-yellow particles (Figure 1).

### 3.5. The Relationship between HER2 Expression and Pathological Features in NSCLC Tissue

As shown in Table 4, the results showed that the positive expression of HER2 was significantly correlated with tumor type, tumor size, tumor differentiation, and lymph node metastasis (*P* < 0.05). Compared with gender and smoking history, there was no significant difference (*P* > 0.05). Among the patients, the proportion of patients with adenocarcinoma, tumor diameter less than 4 cm, well-differentiated, and no lymph node metastasis was higher than that of patients with negative expression of HER2 (*P* < 0.05).

## 4. Discussion

DNMT1 is a maintenance DNA methylation and DNA methyltransferase, which can methylate the corresponding part of DNA semireserved replication in the regenerated strand [9, 10]. Previous study has found that DNMT1 inhibitors play a key role in tumor therapy, suggesting that DNMT1 has a key value in tumor research. Non-small-cell lung cancers such as squamous cell carcinomas, adenocarcinomas, and large cell carcinomas account for a high proportion of lung cancers [11]. Many studies have shown that DNMT1 protein is highly expressed in non-small-cell lung cancer tissues [12, 13].

In this study, we detected serum DNMT1 protein concentrations in lung cancer patients and controls. The results showed that the serum DNMTI protein concentration in the observation group was significantly higher than that in the control group. Gender, age, smoking history, and serum DNMT1 protein concentration were all significantly correlated, indicating that gender, age, and smoking history may be sensitive factors for the high expression of serum DNMT1 protein. Consistent with the results of Zhang et al. [14], the results of this study also suggested that the serum DNMT1 protein concentration of the observation group was related to the clinical histological type and clinical stage. The serum DNMT1 protein concentration of patients with stage I+II was significantly higher than that of stage III+IV. The reason may be related to changes in gene methylation status, as an early event of cell carcinogenesis, which may reflect the histopathological type. The positive expression of HER2 was related to tumor type, tumor size, degree of differentiation, and lymph node metastasis, indicating that the overexpression of HER2 may play important role in advanced NSCLC events. In this study, the correlation between the pathological characteristics and HER2 expression level was investigated. Patients with adenocarcinoma, tumor diameter over 4 cm, poorly differentiated, and lymph node metastasis had a higher degree of HER2 positive expression, indicating that HER2 overexpression mainly occurs in lung adenocarcinoma in advanced patients. Although the current results indicate that HER2 may be difficult to detect as an independent predictor, and other genes need to be combined to detect the occurrence of lung cancer, in terms of prognosis, previous study have shown that the high expression of HER2 is due to the abnormal expression of the normal ErbB2 gene. The ErbB2 gene is an important therapeutic target for NSCLC, so HER2 has a positive significance in predicting the prognosis of patients [15]. Previous study indicated that the tyrosine kinase activity of HER3 is missing, and even if it is combined with a ligand, it cannot activate the downstream signal channel, but it can combine with HER2 to form a dimer with the strongest signaling ability in the family [16]. When the heterodimer is formed, it can also be combined with other ligands, so that it has a variety of activation signals and then regulates cell proliferation, invasion, differentiation, and cell migration through various pathways such as Akt and MAPK. Therefore, the results of this study suggest that in future clinical studies, it is necessary to pay more attention to the high expression of HER2 in tumor patients, in order to grasp the specific information of their disease changes and provide reliable information for the adjustment of clinical treatment plans and the reduction of the incidence of mid- to late-stage events in a timely manner.

In summary, the high expression of DNMT1 serum protein may play a major role in the early development of lung cancer and is a risk factor for non-small-cell lung cancer; the positive expression of HER2 is of great significance to the development of lung cancer in the middle and late stages. The progression of metastatic non-small-cell lung cancer may have a driving effect.

## Figures and Tables

**Figure 1:** HER2 expression in lung cancer and adjacent tissues was determined by immunohistochemistry. Representative images of (a) tissues were collected from NSCLC patients. (b) Samples were collected from the adjacent tissue.

**Table 1:** General information of patients in two groups.

Group	Number of cases	Male/female (example)	Age (years)	Smoking/not smoking
Observation group	60	41/19	61.4 ± 1.6	44/16
Control group	60	39/21	60.3 ± 1.5	46/14
*t*/*χ*^2^	/	12.387	8.943	9.846
*P*	/	0.193	0.084	0.138

**Table 2:** Comparison of DNMT1 protein concentration in serum.

Group		Number of cases	DNMT1 (*μ*g/L)
Observation group	Gender (men and women)	41/19	15.2 ± 10.1^a^/16.3 ± 9.9^a^
	Age (≦60/>60years)	34/26	18.4 ± 10.2^a^/14.4 ± 10.4^a^
	Smoking (yes/no)	44/16	108.5 ± 22.5^a^/107.5 ± 21.0^a^
Control group	Gender (men and women)	39/21	10.5 ± 9/13.2 ± 10.2
	Age (≦60/>60years)	31/29	13.8 ± 10.3/11.3 ± 10.2
	Smoking (yes/no)	46/14	108.3 ± 21.9/105.6 ± 21.1

^a^ *P* < 0.05.

**Table 3:** The relationship between different clinicopathological characteristics of observation group and serum DNMT1 protein concentration.

Pathological features		Number of cases	DNMT1(*μ*g/L)
Histological type	Squamous cell carcinoma	24	29.5 ± 5.1^a^
	Adenocarcinoma	19	26.3 ± 4.2
	Large cell lung cancer	17	27.4 ± 4.2
TNM staging	Phase I+II	34	28.4 ± 5.2^b^
	Phase III+IV	26	27.2 ± 4.5

Note: compared with other histological types, ^a^*P* < 0.05; compared with stage III+IV, ^b^*P* < 0.05.

**Table 4:** Relationship between HER2 expression and pathological characteristics.

Index	HER2	
	*r*	*P*
Gender	0.336	0.241
Smoking history	0.389	0.173
Tumor type	0.497	0.013
Tumor size	0.557	0.002
Tumor differentiation	-0.582	0.001
Lymph node metastasis	0.601	0.000

## Data Availability

The authors confirm that the data supporting the findings of this study are available within the article.
